The article "Botulinum Toxin Type A Injection Improves the Intraperitoneal High Pressure in Rats Treated with Abdominal Wall Plasty" was retracted in 2022. Reason: concerns about the peer review.

# Botulinum Toxin Type A Injection Improves the Intraperitoneal High Pressure in Rats Treated with Abdominal Wall Plasty

**DOI:** 10.1155/2022/1054299

**Published:** 2022-03-15

**Authors:** Xue Zhang, Yingmo Shen, Shuo Yang, Baoshan Wang, Jie Chen

**Affiliations:** Beijing Chaoyang Hospital, Capital Medical University, Beijing, China

## Abstract

The aim of the study is mainly to study the subject of BoNT-A injection to improve IAH in rats undergoing abdominal angioplasty. The study problem in surgery, especially in ICU, burn, and trauma centers, intra-abdominal hypertension (IAH), and abdominal compartment syndrome (ACS) are common complications. At present, there are various treatments for IAH. The intramuscular injection of Botulinum toxin type A (BoNT-A) into the abdominal wall has received a lot of attention. Based on this, this study proposes a method for measuring abdominal pressure, applies BoNT-A to reduce abdominal pressure in the IAH state of abdominal wall angioplasty, and explores a way to increase the compliance of the abdominal wall under the premise of maintaining the sealing of the abdominal cavity, so as to realize the expansion of the abdominal cavity. A method is achieved to reduce intra-abdominal pressure and eliminate or alleviate ACS. The results of the experiment showed that when the rats in the control group were injected with the same amount of normal saline as the rats in the experimental group, the IAP was significantly higher than that in the experimental group (*P* < 0.05). This shows that BoNT-A increases the compliance of the abdominal wall while maintaining the closure of the abdominal cavity, thereby increasing the volume of the abdominal cavity and alleviating the state of IAH in rats.

## 1. Introduction

In recent years, due to the gradual increase in mortality of ACS and IAH, effective treatment of them has attracted increasing attention [1, 2]. So far, abdominoplasty is still an effective measure for the treatment of IAH [3]. The therapeutic botulinum toxin type A is artificially extracted from botulinum toxin type A. The efficacy and safety of BoNT-A injection therapy have been affirmed by the academic community and the industry [4, 5]. Therefore, exploring BoNT-A injection to improve IAH in rats undergoing abdominal angioplasty has important research significance.

Regarding the study of BoNT-A and IAH, many scholars have conducted multiangle explorations. For example, the overactivity of the whole body joints caused by Noonan syndrome leads to children's trapezius spasm and causes neck pain and craniocervical headaches; Tofts LJ studied the effect of BoNT-A on its treatment [6]; Bittar studied the efficacy of BoNT-A in the treatment of postherpetic neuralgia [7]; Park studied the effect of Botox type A through the JNK signaling pathway that inhibits the pro-fibrosis effect of hypertrophic scar fibroblasts [8]. It can be seen that there are few studies on the effect of BoNT-A on IAH in rats. In this paper, BoNT-A injection is used to improve IAH in rats undergoing abdominal angioplasty.

The article "Botulinum Toxin Type A Injection Improves the Intraperitoneal High Pressure in Rats Treated with Abdominal Wall Plasty" was retracted in 2022. Reason: concerns about the peer review.

The study contribution takes IAH as the research object to study the mechanism of BoNT-A on improving IAH in rats undergoing abdominal wall angioplasty. This article first presents a method for detecting abdominal pressure in rats, as well as a model of IAH in an animal. Different doses of BoNT-A were set in the control and experimental groups to evaluate the effect of BoNT-A on decreasing abdominal pressure in the IAH state of abdominal wall angioplasty. BoNT-A can increase abdominal wall compliance while preserving abdominal cavity closure and reduce IAH in rats, according to the results of the experiments.

This study found that injecting BoNT-A into the abdominal wall muscles of rats increased the abdominal cavity's volume and decreased its pressure, providing BoNT-A for the clinical treatment of abdominal compartment syndrome A reliable basis.

## 2. Measurement Design of Intra-Abdominal Pressure in Rats

### 2.1. Making a Simple IAP Meter

Materials needed: desktop sphygmomanometer, disposable infusion set, three-way tube, disposable intravenous infusion needle (0.9 × 28TWLB), 50 ml syringe, nitrogen gas storage bag.

Production method: cut out the infusion tube about 40 cm in length from the disposable infusion set, save one end of the filter, connect the disposable intravenous infusion needle (0.9 × 28TWLB), connect the other end to the tee tube, and unplug the desktop sphygmomanometer, and the connecting tube between the cuffs connects the other ends of the tee tube with the infusion tube to the sphygmomanometer and the other tee tube with a 50 ml syringe and an oxygen bag for storing nitrogen.

### 2.2. IAH Animal Model Preparation

Female/male Sprague Dawley rats are randomly selected weighing about 220 g-250 g. The rats were anesthetized by intraperitoneal injection of 3% pentobarbital sodium (30 mg/kg) to maintain the rats' spontaneous breathing. After the rat is anesthetized successfully, place the rat on the rat board, prepare the skin on both sides of the groin, cut the skin, and routinely disinfect, and then, place a disposable intravenous infusion needle (0.9 × 28TWLB) at a 45-degree angle with the abdominal wall in the left lower abdomen. Slowly puncture the needle toward the upper part of the abdomen and place it into the abdominal cavity. Connect the sphygmomanometer and the nitrogen gas storage bag through the three-way tube, and connect the gas storage bag to a 50 ml syringe. Inject the nitrogen-connected insufficiency needle into the abdominal cavity of the rat, slowly and continuously increase the amount of gas into the abdomen, and continuously monitor IAP dynamically [9].

The article "Botulinum Toxin Type A Injection Improves the Intraperitoneal High Pressure in Rats Treated with Abdominal Wall Plasty" was retracted in 2022. Reason: concerns about the peer review.

### 2.3. Mortality of Rats with Different IAP Levels at Various Time Points

The mortality of rats with different IAP levels at various time points is shown in Table 1: Group 1 rats died within 6 h of IAH and died at 4 different time points of IAH (IAH 1 h, 2 h, 4 h, and 6 h). The change trend of the rate is not obvious. The mortality of rats in the second group showed a gradual upward trend at the above 4 different time points. All 10 rats in the third group died within 2 hours, and 9 of them died within 1 hour.

Figure 1 shows that IAP10 mmHg for more than 2 h can cause abnormal abdominal function and IAP20 mmHg for more than 1 h can cause abnormal abdominal function and cause death. The higher the IAP, the higher the mortality of rats.

## 3. Experimental Design

### 3.1. Experimental Animals

There are 50 Sprague Dawley rats, male and female randomly, weighing about 220 g–250 g. Experimental animals that have been kept in the experimental animal center for at least 7 days were selected. All experimental animals were given free drinking water and granular rat feed according to the standards of the Experimental Animal Center and maintained a light-dark cycle for 12 h–12 h every day. Fasting was carried out for 12 h–16 h before surgery, and there was no restriction on drinking water.

### 3.2. Experiment Grouping and Specific Operations

#### 3.2.1. Group Experiment Setting

Each pair of rats was randomly divided into the experimental group and control group, with 25 rats in each group. After fasting for 8 hours, ketamine hydrochloride injection (100 mg/kg) was used for intraperitoneal anesthesia. After successful anesthesia, the rats were fixed in the supine position on the operating table. After preparing and disinfecting the abdomen, the skin is incised along the midline of the lower abdomen and enters the white line into the abdominal cavity. The incision is about 1.5 cm long. A pressure-measuring balloon and a water injection tube are inserted into the abdominal cavity. The balloon catheter and the water injection tube are fixed on the abdominal wall.

#### 3.2.2. Abdominal Pressure Measurement

The direct pressure measurement method is used for abdominal pressure measurement. During the pressure measurement process, it needs to pay attention to keeping the position of the pressure measurement tube and the pressure sensor at the same level. And the water injection pipe is connected to 500 ml 0.9% sodium chloride warm solution through a disposable infusion set, a small opening is cut on the upper side of the sodium chloride injection infusion bag to ensure that the pressure of the liquid plane is equal to the atmospheric pressure, and the flow regulator is adjusted. The gas in the drip hopper of the infusion set is completely discharged, and the liquid dripping speed is maintained at 40 ml/min. When the pressure in the abdominal cavity of the two groups of rats stabilizes at about 15 mmHg, the flow regulator is closed and the injection of each rat at this time water volume, about 350 ml/kg, is recorded. After completing the measurement, the water is released in the abdominal cavity.

The article "Botulinum Toxin Type A Injection Improves the Intraperitoneal High Pressure in Rats Treated with Abdominal Wall Plasty" was retracted in 2022. Reason: concerns about the peer review.

#### 3.2.3. Inject BoNT-A and Measure Intra-Abdominal Pressure

*(1) Experimental Group*. 0.8 ml of BoNT-A solution was injected into the abdomen of rats in the experimental group, and then, the intra-abdominal water injection tube and balloon piezometer were taken out, and the abdominal incision was sutured. Two days later, when the rats in the experimental group were injected with about 400 ml/kg of normal saline again, the pressure value at this time was less than 15 mmHg, and the water injection was continued to 15 mmHg. At this time, the water injection volume was about 510 ml/kg. The height of the infusion stand is adjusted to make the infusion. The height of the liquid level in the bag is about 20 cm from the height of the rat horizontal plane, and the intra-abdominal pressure is maintained at about 15 mmHg. After 3 hours, the normal saline in the abdominal cavity was released, the water injection tube and balloon piezometer tube in the abdomen were taken out, and the abdominal incision was sutured.

*(2) Control Group*. The control group was injected with the same amount of normal saline at the same point. First, the intra-abdominal pressure is recorded when about 400 ml/kg of normal saline is injected into the abdomen of the control group rat; after 2 days, the intra-abdominal water injection is continued until the total amount reaches 510 ml/kg, records the intra-abdominal pressure at this time, adjusts the height of the infusion stand to keep the intra-abdominal pressure stable, releases the normal saline in the abdominal cavity after 3 hours, takes out the intra-abdominal water injection tube and balloon piezometer, and sutures the abdominal incision.

The rats in the two groups underwent left femoral artery puncture, and blood draw 1 h before the start of the experiment, 3 h after IAH, and 3 h after IAH was removed. 15 rats were randomly selected for blood collection at each time point, and blood was collected about 1.5 ml each time. ELISA method was used to detect the content of superoxide dismutase (SOD) and malondialdehyde (MDA) in rats.

The article "Botulinum Toxin Type A Injection Improves the Intraperitoneal High Pressure in Rats Treated with Abdominal Wall Plasty" was retracted in 2022. Reason: concerns about the peer review.

### 3.3. Statistical Analysis

All data in this experiment are statistically analyzed by GraphPad Prism software, and the experimental results are expressed as mean ± standard deviation (mean ± SD). *T*, *Z*, and heterogeneity test methods are used to verify whether the differences in experimental results are statistical significance.

#### 3.3.1. *T*, *Z* Inspection

Statistical test of combined effect size SE(T): to test whether the combined effect size of multiple independent original studies is statistically significant. The *z* test is a commonly used method, and the calculation method is shown as follows:

(1) $$\begin{array}{c} \text{SE}\left(T\right)=\frac{1}{\sqrt{\sum \mathrm{wi}}}, \end{array}$$

(2) $$\begin{array}{c} \text{z}=\frac{\bar{T}}{\text{SE}\left(T\right)}. \end{array}$$

Among them, Wi represents the weight value of the *i*-th study; $\bar{T}$ represents the combined effect size. The *P* value under the probability of this statistic can be obtained from the z value. When *P* < 0.05, the result is considered to have a significant difference. When *P* > 0.05, it means $\bar{T}$ is not statistically significant.

#### 3.3.2. Heterogeneity Test

The basic idea of this method of testing is that all studies come from the same population, so the true effect is consistent in different studies, and the difference between the observed effect sizes is due to sampling errors. The commonly used test is to calculate the chi-square value; that is, the *Q* test is shown as follows:

(3) $$\begin{array}{c} Q=\sum \mathrm{wi}\left(Ti-\bar{T}\right). \end{array}$$

Among them, Ti represents the effect size of the i-th original study. When the result of the *Q* test is *P* > 0.1, it means that multiple original studies have homogeneity; when the result of the *Q* test is *P* < 0.1, it means that there are multiple original studies, and there is no homogeneity between studies.

### 3.4. Relationship between Intraperitoneal Water Injection and IAP

The comparison results of IAP between the two groups of rats with the same three intraperitoneal injections are shown in Table 2: when the first injection of water, the abdominal pressure of the two groups of rats can reach 12–15 mmHg. During the second water injection, the rats in the experimental group had an average IAP of only 10.72 mmHg; during the third injection, the IAP reached 14.49 mmHg; while in the control group during the second injection, the IAP reached 14.96 mmHg, compared with the experimental group of rats. The difference was statistically significant (*P* < 0.01); when the third water injection, the average IAP reached 17.63 mmHg, and compared with the experimental group of rats, the difference was statistically significant (*P* < 0.01).

The article "Botulinum Toxin Type A Injection Improves the Intraperitoneal High Pressure in Rats Treated with Abdominal Wall Plasty" was retracted in 2022. Reason: concerns about the peer review.

Figure 2 shows that the injection of BoNT-A into the abdominal muscles of rats can effectively reduce IAH. Two days after the rats in the experimental group were injected with BoNT-A intramuscularly, they were injected with the same physiological saline as the first water injection, and the IAP was significantly reduced, indicating that BoNT-A increased the compliance of the abdominal wall while maintaining the sealing of the abdominal cavity. And it can expand the volume of the abdominal cavity and relieve the IAH state of rats.

### 3.5. Comparison of Serum MDA Content

The comparison results of the serum MDA content of the two groups of rats are shown in Table 3.

It can be seen from Table 3 and Figure 3 that the serum MDA content of the two groups of rats was higher than before the establishment of the IAH model (*P* < 0.05) at the two time points of IAH 3 h and 3 h after IAH withdrawal. Moreover, the serum MDA content of rats in the control group increased more than that in the experimental group, and T test of experimental group and control group data *P* < 0.05.

### 3.6. Rat Serum SOD Content

The comparison results of the serum SOD content of the two groups of rats are shown in Table 4: the serum SOD content of the two groups of rats has a significant decrease in the two time points of IAH 3 h and 3 h after IAH withdrawal (*P* < 0.05). Moreover, the serum SOD content of rats in the control group was lower than that in the experimental group (*P* < 0.05).

According to Figure 4, when IAH is maintained for 3 hours and pressure is withdrawn for 3 hours, the serum SOD content of rats in the two experimental groups has a greater decrease, which indicates that the ischemia/reperfusion injury of rats in the experimental group is significantly less than that in the control group. It is said that BoNT-A reduces the ischemia/reperfusion injury while reducing the body's IAH.

## 4. BoNT-A Injection Improves IAH in Rats Undergoing Abdominal Angioplasty

This study found that the two groups of rats had different degrees of peroxidation damage after IAH3h and IAH3h were withdrawn. Compared with the normal abdominal pressure, the two groups of rats also showed increased serum MDA levels (*P* < 0.05) and decreased SOD activity (*P* < 0.05) within the same period of time. The two indicators changed after 3 hours of withdrawal more significantly (*P* < 0.05). This shows that the body has different degrees of ischemia/reperfusion injury during IAH and after decompression.

The article "Botulinum Toxin Type A Injection Improves the Intraperitoneal High Pressure in Rats Treated with Abdominal Wall Plasty" was retracted in 2022. Reason: concerns about the peer review.

IAH may cause pressure on the blood vessels of the abdominal organs and cause ischemic injury. Ischemia can affect vasodilation and defecation. Furthermore, hypoxia may affect the blood perfusion of specific organs in the abdomen, potentially leading to vascular reperfusion and oxidative stress [10, 11] infliction. When the IAH state is relieved, the blood flow of the kidneys increases. The reperfusion of long-term ischemic and hypoxic tissues and organs produces a large number of oxygen-free radicals in a short period of time. As a result, the ischemia/reperfusion injury becomes more serious.

Therefore, the degree of changes in serum MDA and SOD levels will decrease more significantly after IAH is relieved [12].

At the same time, two days after the rats in the experimental group were injected with BoNT-A intramuscularly, they were injected with the same normal saline as the first water injection, and the IAP was significantly reduced while the rats in the control group received the same amount of intra-abdominal injection as the rats in the experimental group. In normal saline, IAP was significantly higher than that in the experimental group. This indicates that BoNT-A can increase the compliance of the abdominal wall under the premise of keeping the abdominal cavity closed, thereby increasing the abdominal cavity volume and helping to alleviate the state of IAH in rats.

## 5. Conclusion

This study found that BoNT-A injection into the abdominal wall muscles of rats increased the capacity of the abdominal cavity and reduced the pressure of the abdominal cavity, consequently eliminating or easing abdominal compartment syndrome. The foundation is solid. As a result, injecting BoNT-A into the abdomen wall intramuscularly to prevent and treat IAH has a favorable impact on lowering intra-abdominal pressure and can be utilized in clinical IAH therapy.

## Figures and Tables

**Figure 1:** The mortality of rats with different IAP levels at various time points (%).

**Figure 2:** Comparison of IAP when three intraperitoneal water injections are equal (mmHg).

**Figure 3:** Comparison of serum MDA concentration in two groups of rats (nmol/L).

**Figure 4:** Comparison of serum SOD content in the two groups of rats (ng/ml).

**Table 1:** The mortality of rats with different IAP levels at various time points (%).

Sequence	Group	N	Time			
			1 h	2 h	4 h	6
IAP10 mmHg	1	10	0	0	0	20%
IAP15 mmHg	2	10	20%	40%	50%	75%
IAP20 mmHg	3	10	90%	100%	—	—

**Table 2:** Comparison of IAP when three intraperitoneal water injections are equal (mmHg).

Animal grouping	*N*	Time		
		The 1st time	The 2nd time	The 3rd time
Test group	15	12.19 ± 0.43	10.72 ± 0.67^*∗*^	14.49 ± 0.22^*∗*^
Control group	15	14.74 ± 0.27	14.96 ± 0.54	17.63 ± 0.64

(Note: ^*∗*^*P* < 0.01, ^#^*P* < 0.05).

The article "Botulinum Toxin Type A Injection Improves the Intraperitoneal High Pressure in Rats Treated with Abdominal Wall Plasty" was retracted in 2022. Reason: concerns about the peer review.

**Table 3:** Comparison of serum MDA concentration in two groups of rats (nmol/L).

Grouping	*N*	Time		
		1 h before surgery	IAH 3 h	IAH decompression 3 h
Test group	15	0.77 ± 0.24	1.32 ± 0.41^*∗*^#	1.63 ± 0.47^*∗*^#
Control group	15	0.81 ± 0.22	1.55 ± 0.67#	2.17 ± 0.24#

(Note: compared with the control group, ^*∗*^*P* < 0.05, and compared with preoperatively, ^#^*P* < 0.05)

**Table 4:** Comparison of serum SOD content in the two groups of rats (ng/ml).

Grouping	*N*	Time		
		1 h before surgery	IAH3 h	IAH decompression 3 h
Test group	10	88.07 ± 18.06	83.04 ± 3.52^*∗*^#	63.02 ± 4.05^*∗*^#
Control group	10	88.07 ± 18.06	70.90 ± 3.20#	47.61 ± 3.21#

Note. Compared with the control group, ^*∗*^*P* < 0.05; compared with preoperatively, ^#^*P* < 0.05.

## Data Availability

The data underlying the results presented in the study are available within the manuscript.

## References

[1] Skervin A., Mobasheri M. (2019). Abdominal compartment syndrome. *Surgery*.

[2] di Natale A., Moehrlen U., Neeser H. R. (2020). Abdominal compartment syndrome and decompressive laparotomy in children: a 9 year single-center experience. *Pediatric Surgery International*.

[3] Sun J., Sun H., Sun Z., Xin Y., Shuhua Z., Jianxin W. (2021). Intra-abdominal hypertension and increased acute kidney injury risk: a systematic review and meta-analysis. *Journal of International Medical Research*.

[4] Wang Z. M., Wang Z. Y., Wei C. J., Jia Y. J. (2020). Can Botulinum Toxin Type A effectively treat neuropathic pain in spinal cord injury?: a protocol of systematic review and meta-analysis. *Medicine*.

[5] Colosimo C., Charles D., Charles D. (2019). How satisfied are cervical dystonia patients after 3 years of botulinum toxin type A treatment? Results from a prospective, long-term observational study. *Journal of Neurology*.

[6] Tofts L. J., Waugh M. C., Hayden S. (2019). Effect of Botulinum Toxin type-A (Botox) on neck pain and craniocervical headaches caused by trapezius spasm in a child with generalised joint hypermobility resulting from Noonan’s Syndrome. *Pediatric Rheumatology*.

[7] Bittar J., Ditre C. (2019). Treatment of postherpetic neuralgia with botulinum toxin type A. *Journal of the American Academy of Dermatology*.

[8] Park G. S., An M. K., Yoon J. H. (2019). Botulinum toxin type A suppresses pro-fibrotic effects via the JNK signaling pathway in hypertrophic scar fibroblasts. *Archives of Dermatological Research*.

[9] Kothapalli A., Caccetta T. (2019). Botulinum toxin type A for the first-line treatment of Hailey-Hailey disease. *Australasian Journal of Dermatology*.

The article "Botulinum Toxin Type A Injection Improves the Intraperitoneal High Pressure in Rats Treated with Abdominal Wall Plasty" was retracted in 2022. Reason: concerns about the peer review.

[10] Sousa E. D. J. S. D., Sousa G. C. D., Baia V. F., Somensi D. N., Xavier M. B. (2019). Botulinum toxin type A in chronic neuropathic pain in refractory leprosy. *Arquivos de Neuro-Psiquiatria*.

[11] Oral A. (2020). Is botulinum toxin type A efficacious, safe, and tolerable in cervical dystonia?: a cochrane review summary with commentary. *American Journal of Physical Medicine & Rehabilitation*.

[12] Ismail S. A., Mohammed N., Sotohy M., Taleb D. A. E. A. (2020). Botulinum toxin type A versus 5-Fluorouracil in treatment of keloid. *Archives of Dermatological Research*.

